The article "Integrated Learning: Screening Optimal Biomarkers for Identifying Preeclampsia in Placental mRNA Samples" was published in 2021. Journal: Comput Math Methods Med.

# Integrated Learning: Screening Optimal Biomarkers for Identifying Preeclampsia in Placental mRNA Samples

**DOI:** 10.1155/2021/6691096

**Published:** 2021-02-23

**Authors:** Rong Guo, Zhixia Teng, Yiding Wang, Xin Zhou, Heze Xu, Dan Liu

**Affiliations:** ^1^Information and Computer Engineering College, Northeast Forestry University, Harbin 150040, China; ^2^Department of Gynecology and Obstetrics, Tongji Hospital, Tongji Medical College, Huazhong University of Science and Technology, Wuhan, Hubei, China

## Abstract

Preeclampsia (PE) is a maternal disease that causes maternal and child death. Treatment and preventive measures are not sound enough. The problem of PE screening has attracted much attention. The purpose of this study is to screen placental mRNA to obtain the best PE biomarkers for identifying patients with PE. We use Limma in the R language to screen out the 48 differentially expressed genes with the largest differences and used correlation-based feature selection algorithms to reduce the dimensionality and avoid attribute redundancy arising from too many mRNA samples participating in the classification. After reducing the mRNA attributes, the mRNA samples are sorted from large to small according to information gain. In this study, a classifier model is designed to identify whether samples had PE through mRNA in the placenta. To improve the accuracy of classification and avoid overfitting, three classifiers, including C4.5, AdaBoost, and multilayer perceptron, are used. We use the majority voting strategy integrated with the differentially expressed genes and the genes filtered by the best subset method as comparison methods to train the classifier. The results show that the classification accuracy rate has increased from 79% to 82.2%, and the number of mRNA features has decreased from 48 to 13. This study provides clues for the main PE biomarkers of mRNA in the placenta and provides ideas for the treatment and screening of PE.

## 1. Introduction

Preeclampsia (PE) is a pregnancy-specific syndrome that affects 3-5% of pregnant women and is characterized by edema, hypertension, and proteinuria [1]. PE is a multifactor and multigene disease with a family genetic predisposition: assuming a mother had PE, the incidence of PE in her daughters is 20-40%. If a twin is a patient with PE, the incidence of PE in the other twin is 22-47%. PE makes women more susceptible to cardiovascular disease later in life and may affect brain function. However, so far, the genetic pattern is unclear. It remains a major factor in maternal and newborn morbidity and mortality [2]. The only treatment is the termination of pregnancy and delivery of newborns and the placenta [3]. Although the causes of PE are still being discussed, clinical and pathological studies have shown that the core of the pathogenesis of this syndrome is the placenta [4]. The placenta is an important organ shared by the mother and the fetus. It has important biological functions such as substance exchange, metabolism, and barrier function. Abnormal placental function can lead to pregnancy diseases such as PE. Many physiological and biochemical processes related to placental function are coordinated by proteins that form complex networks in the placenta, and the production of proteins requires the participation of RNA.

In the study of the biomarkers of PE, genetic factors were found to be the cause of the disease [5]. In naive Bayesian predictive modeling and path analysis, the quantitative real-time polymerase chain reaction (qRT-PCR) concluded that genes in the placenta are related to PE through genetic testing [6]. The genetic markers of normal fluff in the placenta can express pathology and PE [7]. Clinically relevant subcategories are identified by the gene expression profile of the placenta [8].

However, research on mRNA in the placenta that can be used as a biomarker for PE is still insufficient. mRNA is a direct template for directing protein synthesis, that is, transferring genetic information from DNA to RNA. mRNA is used as a template for protein synthesis to determine the amino acid sequence of the peptide chain produced by gene expression proteins, and proteins such as VEGF, sFlt1, PlGF, SENG, PAPP-A, PP13, HSP70, and HbF have shown certain value in the prediction or diagnosis of PE [9] (review). This helps in the understanding of the pathogenesis of PE. In these studies, it can be inferred that an abnormal expression of mRNA in the placenta is related to the occurrence of PE, and there are mRNA samples that can be used to identify PE.

Traditional medical methods generally can find only a few biomarkers, and the accuracy of disease recognition is difficult to guarantee. Machine learning performs well in feature filtering and processing large amounts of data [10] (review) and performs well in RNA research [11, 12]. In this study, classification algorithms can be used to detect the mRNA biomarkers of PE in the placenta and to screen out the mRNA samples that can be used as biomarkers in the dataset to avoid the omission of biomarkers. By fusing multiple classifiers, the accuracy of the algorithm is improved, and overfitting is reduced.

## 2. Materials and Methods

### 2.1. Data Source

The GSE75010 dataset used in the experiment is the placental microarray dataset released on May 16, 2016, for the analysis of placental gene expression profiles. It is a large dataset containing data from seven published studies (*N* = 330) [13]. This dataset was downloaded from the GEO database and contains gene expression data from 157 placentas with PE and 173 placentas without PE. For convenience, we choose 157 highly annotated samples as the experimental dataset to model and test the classification effect.

### 2.2. Identification of Differentially Expressed Genes

To standardize the microarray data [14], the GSE75010 dataset downloaded from the GEO database was converted to log2 with the Limma package in R3.4.1. The dataset is divided into two categories according to disease status: placenta with PE and healthy control placenta. The two sets of gene expression matrices were compared by the Limma package [15], and the thresholds were set to |logFC| > 2 and *P* < 0.01.

### 2.3. Feature Selection

Correlation-based feature selection (CFS) [16] is a heuristic algorithm based on filter patterns. It can improve the classification effect by evaluating the correlation among features as well as the correlation between features and categories. It finds the optimal subset of features to avoid redundancy among the features. Differentially expressed mRNA samples do not necessarily belong to the mRNA samples related to PE. The purpose of CFS is to exclude irrelevant differential genes while avoiding too many mRNA samples participating in the classification, thereby improving the accuracy of classification.

(1) $$\begin{array}{c} {\text{Merit}}_{s}=\frac{k\bar{r_{cf}}}{\sqrt{k+k\left(k-1\right)\bar{r_{ff}}}}. \end{array}$$

*k* represents the number of features in the subset, $\bar{r_{cf}}$ represents the average correlation between features and categories, and $\bar{r_{ff}}$ represents the average correlation among features. The Pearson correlation coefficient [17] is used to calculate $\bar{r_{cf}}$ and $\bar{r_{ff}}$ and can be used to measure the correlation between two variables and screen out mRNA samples related to PE.

(2) $$\begin{array}{c} r\left(X,Y\right)=\frac{\sum_{1}^{n}\left(X_{i}-\bar{X}\right)\left(Y_{i}-\bar{Y}\right)}{\sqrt{\sum_{1}^{n}{\left(X_{i}-\bar{X}\right)}^{2}{\left(Y_{i}-\bar{Y}\right)}^{2}}}. \end{array}$$

To improve the classification efficiency of the optimal subset, the information gain ratio algorithm is used to sort the mRNA samples in the optimal subset from large to small [18]. It enables the classifier to classify according to the amount of mRNA information, thereby improving the accuracy of classification. This is an algorithm developed by information entropy. The formula is as follows:

(3) $$\begin{array}{c} \text{Ent}\left(D\right)=-\overset{\left|y\right|}{\underset{k=1}{\sum }}p_{k}\log_{2}p_{k}. \end{array}$$

|*y*| represents the number of categories *p*_*k*_, which is the proportion of each category feature in the set. The result of this formula represents the entropy of the information carried by mRNA [19]. The smaller the information entropy is, the purer the dataset.

The value of information gain [20] can determine whether to use this mRNA attribute *a* to divide dataset *D*. If the information gain is relatively large, this attribute is a better attribute for dividing dataset *D*.

(4) $$\begin{array}{c} \text{Gain}\left(D,a\right)=\text{Ent}\left(D\right)-\overset{V}{\underset{v=1}{\sum }}\frac{\left|D^{v}\right|}{\left|D\right|}\text{Ent}\left(D^{v}\right). \end{array}$$

Information gain is biased towards selecting features with more values in the same category, but according to the entropy formula, the more features there are, the greater the entropy is. To change the adverse effects of such poor preferences, this study uses the information gain ratio [21] as a method to judge the division of attributes.

(5) $$\begin{array}{c} \text{Gain}\_\text{ratio}\left(D,a\right)=\frac{\text{Gain}\left(D,a\right)}{-\sum_{v=1}^{V}\left|D^{v}\right|/\left|D\right|\log_{2}\left|D^{v}\right|/\left|D\right|} \end{array}$$

Finally, according to the results of mRNA information gain, we sorted the mRNA samples in the optimal subset from largest to smallest to train the classifier. On the one hand, the information gain ratio can be a measure of the importance of mRNA, and on the other hand, it can be used as a node selection criterion for the C4.5 classifier.

### 2.4. Classification Algorithm Design

After filtering mRNA as a feature through the above algorithm, to facilitate sample classification, we designed a suitable model. The trained model can use mRNA samples as attributes to identify whether pregnant women have PE. The disadvantage of small sample datasets is that they are easy to overfit during classification, and ensemble learning is one of the basic methods to alleviate this situation to some extent. We chose three different classifiers as subclassifiers.

Subclassifier I is a C4.5 [22] decision tree that selects attributes according to the information gain ratio and has a good classification effect on small sample datasets. To improve operation efficiency, this C4.5 decision tree is generated in the form of a binary tree.

Subclassifier II is a multilayer perceptron [23]. The multilayer perceptron continuously updates the weights through the backpropagation (BP) algorithm. A learning rate that is too low can greatly increase the training time of the model, and a learning rate that is too large can cause underfitting, so the learning rate is set to 0.3. When the standard BP algorithm corrects the weights, a momentum factor is added to each weight change to prevent the multilayer perceptron from falling into a local minimum, and the momentum factor is set to 0.2. The momentum factor value is the opposite of the value of the last weight change, thus affecting the new weight change based on the BP method. The number of mRNA attributes is set to the number of nodes in the hidden layer, the number of training iterations is initialized to 500, and the network is reset at a lower learning rate. If the network deviates from the answer, it will automatically reset and retrain at a lower learning rate.

(6) $$\begin{array}{c} S\left(x\right)=\frac{1}{1+e^{-x}}. \end{array}$$

The network maps each data point to an interval (0,1) or (-1,0) to achieve the effect of classification.

Subclassifier III is a decision stump [24] integrated by AdaBoost [25]. The AdaBoost algorithm modifies the classifier and sample weights by continuously iterating the training dataset and integrating many weak classifiers into a strong classifier, as shown in the following formula:

(7) $$\begin{array}{c} F\left(x\right)=\overset{T}{\underset{t=1}{\sum }}\alpha_{t}f_{t}\left(x\right). \end{array}$$

*T* represents the number of weak classifiers, *α*_*t*_ represents the weight of the *t*-th weak classifier, and *f*_*t*_(*x*) represents the prediction result of the *t*-th weak classifier. The final classification decision rules are as follows:

(8) $$\begin{array}{c} \mathrm{sgn}\left(F\left(x\right)\right)=\left\{\begin{array}{c} 1,x>0,\\ -1,x<0. \end{array}\right. \end{array}$$

Finally, we use majority voting to integrate subclassifiers. This is an ensemble method that uses most of the output results of the subclassifiers as the final classification result. All models and algorithms are built into Weka 3.8.4 [26].

### 2.5. Evaluation Criteria

Cross validation (CV) [27, 28], sometimes called rotation estimation, is a statistical method proposed by Seymour Geisser to cut data samples into smaller subsets. For small sample data, CV can avoid overfitting to a certain extent, making the training model more versatile, robust, and accurate. This experiment uses a 10-fold CV method to train the model, that is, the dataset is divided into ten parts, each of which uses 9 different parts for training and one to verify the model to ensure that all the datasets are tested. The idea of tenfold CV is shown in Figure 1.

To facilitate the discussion below, we set the placentas with PE as positive samples and the healthy placentas as negative samples. We use the following indicators as the criteria for evaluating the classifier [29–35]:

(9) $$\begin{array}{c} \text{Recall}=\frac{\text{TP}}{\text{TP}+\text{FN}},\\ \text{Precision}=\frac{\text{TP}}{\text{TP}+\text{FP}},\\ \text{Accuracy}=\frac{\text{TP}+\text{TN}}{\text{TP}+\text{TN}+\text{FP}+\text{FN}},\\ \text{Specificity}=\frac{\text{TN}}{\text{TN}+\text{FP}},\\ \text{Sensitivity}=\frac{\text{TP}}{\text{TP}+\text{FN}}. \end{array}$$

Specificity and sensitivity are both indicators of successful model classification. Specificity is an indicator that measures the probability of diagnosis, and sensitivity is an indicator that measures the recognition ability of a classification model. We also introduced the area under the curve (AUC) as an indicator to measure the effectiveness of the model. The AUC is the area between the receiver operating curve (ROC) and the coordinate axis. Its value is in the interval (0.5,1). The closer the AUC value is to 1, the better the classifier is.

## 3. Results and Discussion

The results of the differential gene analysis are represented by a volcano plot in Figure 2(green indicates a relatively low mRNA expression, red indicates relatively high mRNA expression, and gray indicated undifferentiated mRNA samples).

Figure 3 below shows the relative expression levels of the 48 differential genes screened by Limma in the preeclamptic placenta, denoted in the figure as PE, and the control healthy placenta, denoted in the figure as control (green indicates relatively low mRNA expression and red indicates relatively high mRNA expression).

After screening out 48 differential genes, CFS was used to filter mRNA to remove irrelevant mRNA and redundant mRNA. The optimal subset consisting of 13 mRNA attributes was obtained (HTRA4, PROCR, MYCN, ERO1A, EAF1, PPP1R16B, CRH, FLNB, PIK3CB, PLAAT3, FBN2, RFLNB, and TKT). The results, sorted from largest to smallest by the information gain ratio, were PIK3CB, HTRA4, ERO1A, PPP1R16B, PROCR, CRH, FLNB, PLAAT3, FBN2, EAF1, TKT, RFLNB, and MYCN. In the table, PE represents a sample of patients with PE, control represents a sample of healthy pregnant women as a control group, and average represents the average of the two sets of data. The classification results are derived from mRNA samples in the best subset training model (see Table 1).

Next, we used 48 differentially expressed mRNA samples that were not processed by CFS (the original differentially expressed mRNA samples) to train the model and test the classification effect. The results are as follows (see Table 2):

Table 2 shows that the likelihood of a sample being correctly classified as PE is 0.763, and the accuracy of the overall classification results of the model is 0.790.

By comparing the results from the two sets of experiments, it can be seen that the accuracy of the optimal subset of mRNA is 0.822, in which the correctly classified PE samples have increased from 61 to 63, and the correctly classified control samples have increased from 63 to 66.

However, it is not comprehensive to select the best biomarkers based on classification accuracy alone. We also use recall, precision, and AUC as classification criteria to obtain more comprehensive results.

Notably, recall, precision, and AUC reached the maximum values in Table 1; the specificity increased from 0.818 to 0.857, and the sensitivity increased from 0.763 to 0.788 (see Table 3), which can be considered as high specificity and sensitivity.

In the study of PE, the positive accuracy of the biomarkers discovered by Zeisler et al. was no more than 50% [36], and the positive accuracy of the mRNA PE biomarkers we screened for reached 0.788.

The experiments show that the use of CFS filtering attributes is also applicable to mRNA. After reducing the mRNA dimension, all indicators that have a positive significance for the classification effect are improved.

In the research of Mehmood et al., the voting integration method and the CFS algorithm were also used to achieve ideal results. Although similar algorithms on different datasets may have very different results, for this experiment, the CFS algorithm can exclude irrelevant differential genes, can avoid the redundancy of related mRNA samples, and can maintain the maximum independence among attributes, which is necessary for our research [37].

In this study, the use of the information gain ratio to analyze differential genes can allow for the measurement of the amount of information that mRNA carries for disease outcomes. A variety of classification algorithms are used to test the association between mRNA and PE, and we used placental mRNA to identify PE. Analyses and comparisons were also conducted.

We analyzed mRNA with the highest information gain ratio in the best subset through the Kyoto Encyclopedia of Genes and Genomes (KEGG) pathway, and the results showed that the expression of mRNA (PIK3CB and OCRL) is related to the inositol phosphate metabolism and the phosphatidylinositol signaling systems. This may be related to the biochemical process of PE.

## 4. Conclusions

In recent years, in the classification and screening of genes, it has often only been possible to obtain a single result through differential gene expression analysis. Although this result might be related to PE, the diagnostic effect may not be good enough. However, with the development of machine learning, the use of feature engineering can better improve the classification efficiency, and the use of an appropriate classification model can intuitively reflect the classification effect and indirectly reflect the advantages and disadvantages of attribute selection. Therefore, after analyzing the differentially expressed genes, to improve the classification effect, we used a feature selection algorithm based on correlations as the standard for dimensionality reduction. To obtain better results, we designed a classification model based on a voting mechanism to address the features of small sample datasets that are prone to overfitting. Finally, we used 13 mRNA samples as attributes to obtain satisfactory results. When training the model, we used 10-fold CV to enhance the robustness of the model.

The results show that an accuracy of 82.2% is achieved by the 13 mRNA samples screened out, and the specificity and sensitivity reach 0.857 and 0.788, respectively. The recall of the model is 0.822, the precision is 0.824, and the AUC value reaches 0.822. These indicators reflect that the model has good robustness and a certain generalization ability.

Through the KEGG analysis of the genes in Table 1, PIK3CB and OCRL were found to be involved in the phosphoinositide metabolism and the silanol phosphatidylinositol signaling systems. This can explain the cause of PE from one angle and provide clues for the future treatment of PE.

The optimal subset selected by the CFS algorithm is evaluated by the Pearson coefficient, but the Pearson coefficient cannot screen out important mRNA samples that are nonlinearly related to PE. How to select the optimal subset of mRNA samples that contain nonlinear correlations is still under discussion.

## Figures and Tables

**Figure 1:** 10-fold cross-validation method.

**Figure 2:** Volcano plot of GSE75010.

**Figure 3:** Heatmap of GSE75010.

**Table 1:** Results and indicators of attribute classification (the optimal subset).

	TP/TN	FP/FN	Precision	Recall	AUC
PE	0.788	0.143	0.851	0.788	0.822
Control	0.857	0.213	0.795	0.857	0.822
Average	0.822	0.177	0.824	0.822	0.822

**Table 2:** Results and indicators of attribute classification (the original differentially expressed mRNA samples).

	TP/TN	FP/FN	Precision	Recall	AUC
PE	0.763	0.182	0.813	0.763	0.790
Control	0.818	0.238	0.768	0.818	0.790
Average	0.790	0.209	0.791	0.790	0.790

**Table 3:** Specificity and sensitivity of the original differentially expressed mRNA samples (original) and optimal subset (optimal).

	Specificity	Sensitivity
Original	0.818	0.763
Optimal	0.857	0.788

## Data Availability

The PE dataset in this study can be downloaded from https://www.ncbi.nlm.nih.gov/geo/.

## References

[1] Filipek A., Jurewicz E. (2018). Preeclampsia - a disease of pregnant women. *Postepy Biochemii*.

[2] Landau R., Irion O. (2005). Recent data on the physiopathology of preeclampsia and recommendations for treatment. *Revue Médicale Suisse*.

[3] Bokslag A., van Weissenbruch M., Mol B. W., de Groot C. J. M. (2016). Preeclampsia: short and long-term consequences for mother and neonate. *Early Human Development*.

[4] Rana S., Lemoine E., Granger J. P., Karumanchi S. A. (2019). Preeclampsia: pathophysiology, challenges, and perspectives. *Circulation Research*.

[5] PridjianG P. J. B. (2002). Preeclampsia.Part2: experimental and genetic considerations. *Obstetrical & Gynecological Survey*.

[6] Founds S. A., Conley Y. P., Lyons Weiler J. F., Jeyabalan A., Hogge W. A., Conrad K. P. (2009). Altered global gene expression in first trimester placentas of women destined to develop preeclampsia. *Placenta*.

[7] Leavey K., Benton S. J., Grynspan D., Bainbridge S. A., Morgen E. K., Cox B. J. (2017). Genemarkers of normal villous maturation and their expression in placentas with maturational pathology. *Placenta*.

[8] Leavey K., Benton S. J., Grynspan D., Kingdom J. C., Bainbridge S. A., Cox B. J. (2016). Unsupervised placental gene expression profiling identifies clinically relevant subclasses of human preeclampsia. *Hypertension*.

[9] He A., Zhou Y., Wei Y., Li R. (2020). Potential protein biomarkers for preeclampsia. *Cureus*.

[10] Mirza B., Wang W., Wang J., Choi H., Chung N. C., Ping P. (2019). Machine learning and integrative analysis of biomedical big data. *Genes*.

[11] Sagar A., Xue B. (2019). Recent advances in machine learning based prediction of RNA-protein interactions. *Protein and Peptide Letters*.

[12] Goksuluk D., Zararsiz G., Korkmaz S. (2019). LSeq: machine learning interface for RNA-sequencing data. *Computer Methods and Programs in Biomedicine*.

[13] Leavey K., Wilson S. L., Bainbridge S. A., Robinson W. P., Cox B. J. (2018). Epigenetic regulation of placental gene expression in transcriptional subtypes of preeclampsia. *Clinical Epigenetics*.

[14] Smyth G. K. (2005). Limma: linear models for microarray data. *Bioinformatics and computational biology solutions using R and Bioconductor, Statistics for Biology and Health*.

[15] Ritchie M. E., Phipson B., Wu D. (2015). Limma powers differential expression analyses for RNA-sequencing and microarray studies. *Nucleic Acids Research*.

[16] Ranjan B., Sun W., Park J. (2020). *DUBStepR: correlation-based feature selection for clustering single-cell RNA sequencing data*.

[17] Song J., Liu Y. D., Su J., Yuan D., Sun F., Zhu J. (2019). Systematic analysis of alternative splicing signature unveils prognostic predictor for kidney renal clear cell carcinoma. *Journal of Cellular Physiology*.

[18] Dai J., Xu Q. (2013). Attribute selection based on information gain ratio in fuzzy rough set theory with application to tumor classification. *Applied Soft Computing*.

[19] Monaco A., Pantaleo E., Amoroso N. (2021). Identifying potential gene biomarkers for Parkinson’s disease through an information entropy-based approach. *Physical Biology*.

[20] Batur C., Diri B. Sequence classification based on information gain feature groups using ensemble gene selection framework.

[21] Ghasemi F., Neysiani B. S., Nematbakhsh N. Feature selection in pre-diagnosis heart coronary artery disease detection: a heuristic approach for feature selection based on information gain ratio and Gini index.

[22] Zhou Z.-H., Jiang Y. (2003). Medical diagnosis with C4. 5 rule preceded by artificial neural network ensemble. *IEEE Transactions on Information Technology in Biomedicine*.

[23] Yun J., Park J. E., Lee H., Ham S., Kim N., Kim H. S. (2019). Radiomic features and multilayer perceptron network classifier: a robust MRI classification strategy for distinguishing glioblastoma from primary central nervous system lymphoma. *Scientific Reports*.

[24] Dawngliani M. S., Chandrasekaran N., Lalmawipuii R., Thangkhanhau H., Pandian A., Palanisamy R., Ntalianis K. (2019). Comparison of Decision Tree-Based Learning Algorithms Using Breast Cancer Data. *Proceeding of the International Conference on Computer Networks, Big Data and IoT (ICCBI - 2019). ICCBI 2019. Lecture Notes on Data Engineering and Communications Technologies, vol 49*.

[25] Huang Q., Chen Y., Liu L., Tao D., Li X. (2019). On combining biclustering mining and AdaBoost for breast tumor classification. *IEEE Transactions on Knowledge and Data Engineering*.

[26] Maheshwari A., Chakrabarti P. (2020). Machine learning classifier and neural modelling perspective of echocardiography for thalassemia patients in context to pediatric age group. *Journal of Critical Reviews*.

[27] Ying X. (2019). An overview of overfitting and its solutions. *Journal of Physics: Conference Series*.

[28] Peterson R. A., Cavanaugh J. E. (2020). Ordered quantile normalization: a semiparametric transformation built for the cross-validation era. *Journal of Applied Statistics*.

[29] Min X., Li M., Dong D. (2019). Multi-parametric MRI-based radiomics signature for discriminating between clinically significant and insignificant prostate cancer: cross-validation of a machine learning method. *European Journal of Radiology*.

[30] d’Abramo C., D’Adamio L., Giliberto L. (2020). Significance of blood and cerebrospinal fluid biomarkers for Alzheimer’s disease: sensitivity, specificity and potential for clinical use. *Journal of Personalized Medicine*.

[31] Deng Y., Xu X., Qiu Y., Xia J., Zhang W., Liu S. (2020). A multimodal deep learning framework for predicting drug-drug interaction events. *Bioinformatics*.

[32] Zhang W., Li Z., Guo W., Yang W., Huang F. (2019). A fast linear neighborhood similarity-based network link inference method to predict microRNA-disease associations. *IEEE/ACM Transactions on Computational Biology and Bioinformatics*.

[33] Zhang W., Jing K., Huang F. (2019). SFLLN: a sparse feature learning ensemble method with linear neighborhood regularization for predicting drug–drug interactions. *Information Sciences*.

[34] Zhao Y., Wang F., Chen S., Wan J., Wang G. (2017). Methods of microRNA promoter prediction and transcription factor mediated regulatory network. *BioMed Research International*.

[35] Cheng L., Wang P., Tian R. (2019). LncRNA2Target v2.0: a comprehensive database for target genes of lncRNAs in human and mouse. *Nucleic Acids Research*.

[36] Zeisler H., Llurba E., Chantraine F. (2016). Predictive value of the sFlt-1:PlGF ratio in women with suspected preeclampsia. *The New England Journal of Medicine*.

[37] Mehmood Y., Ishtiaq M., Tariq M., Jaffar M. A. Classifier ensemble optimization for gender classification using genetic algorithm.

